The article "Design of Semiautomatic Digital Creation System for Electronic Music Based on Recurrent Neural Network" was published in 2022. Journal: Comput Intell Neurosci.

# Design of Semiautomatic Digital Creation System for Electronic Music Based on Recurrent Neural Network

**DOI:** 10.1155/2022/5457376

**Published:** 2022-06-27

**Authors:** Yonghui Duan, Jianping Wang

**Affiliations:** ^1^School of Music and Dance of Changzhi University, Changzhi, Shanxi 046011, China; ^2^Department of Intelligence and Automation of Taiyuan University, Taiyuan, Shanxi 030032, China

## Abstract

Semiautomated digital creation is increasingly important in the manipulation of electronic music. How to realize the learning of local effective features of audio data is a difficult point in the current research field. Based on recurrent neural network theory, this paper designs a semiautomatic digital creation system for electronic music for digital manipulation and genre classification. The recurrent neural network improves the transmission of electronic music information between the input and output of the network by adopting dense connections consistent with DenseNet and adopts an inception-like structure for the autonomous selection of effective recursive nuclear electronic music categories. In the simulation process, the prediction method based on semiautomatic digital audio clips is also adopted, which pays more attention to the learning of local effective features of audio data, which gives the model the ability to create audio samples of different lengths and improves the model's support for creative tasks in different scenarios. It includes the determination of the number of neurons, the selection of the function of neurons, the determination of the connection method, and the specific learning algorithm rules, and then the training samples are formed. The experimental results show that the recurrent neural network exhibits powerful feature extraction ability and classification ability of music information. The 10-fold cross-validation on GTZAN dataset and ISMIR2004 dataset has obtained 88.7% and 87.68%, surpassing similar ones. The model has reached a leading level. After further use of the MSD (Million Song Dataset) dataset for pre-semiautomatic training, the model effect has been further greatly improved. The accuracy rate on the dataset has been increased to 91.0% and 89.91%, respectively, which has improved the semiautomatic number and creative advancement.

## 1. Introduction

With the rapid development of Internet technology and digital multimedia technology in recent years, there has been an explosive growth in the number of various artistic works such as literature, photography, and music. More and more people have begun to participate in the creation, dissemination, and appreciation of these works of art through the Internet. For one type of music in these works of art, various types of online music services have become the main channels for people to listen to music on a daily basis [1]. People's personal preferences for genres of musical compositions also drive service providers to provide more accurate music classification results. The traditional way of understanding music and performing recursive classification mainly by professionals is unable to cope with the massive amount of music, and it is imperative to use computer programs to automatically classify music genres [2–5]. In the task of music genre classification, many classical machine learning methods have achieved good results on standard datasets, but these methods make extensive use of recursive features designed by domain experts, and the threshold for non-domain experts is high. Some features lack generality and cannot be well transferred to other fields. With the widespread use of deep learning models in other fields, methods of using deep learning models have also begun to appear in music genre classification tasks [6–9].

The article "Design of Semiautomatic Digital Creation System for Electronic Music Based on Recurrent Neural Network" was published in 2022. Journal: Comput Intell Neurosci.

In music signal processing, recurrent neural network plays a pivotal role, and signal correlation, filtering, and spectral estimation must be realized by discrete Fourier transform. However, when *N* is very large, it is necessary to complete N × *N* complex multiplications and *N*(*N* − 1) complex additions to find a DFT of *N* points, which requires a considerable amount of calculation. Since the original audio data contains sampling frequency, quantization precision, and the limited registration information such as encoding methods, it is only a non-semantic symbolic representation and an unstructured binary stream, lacking content semantic description and structured organization, so applications such as audio recognition, retrieval, and content filtering are all affected limitation [10]. How to extract the structured information and content semantics in the audio, so that the disordered audio data becomes orderly, is the key to whether the content-based audio retrieval technology can be practical. Waveforms have their own characteristics [11–15]. For example, speech audio has the characteristics of large changes and high frequency components because its components are speech; music audio waveforms are relatively smooth and have high frequency components. The characteristics of speech and music frequency waveforms are as follows: high-frequency components have strong energy, the waveform has a certain trend, and it is easier to see the speech components. These characteristics are easy to be identified by people and only need to be rooted on the computer. Basic signal characteristics can classify them.

The article "Design of Semiautomatic Digital Creation System for Electronic Music Based on Recurrent Neural Network" was published in 2022. Journal: Comput Intell Neurosci.

For benchmark model through comparative experiments, this paper proves the positive correlation of pitch features for recognition and explores the number of harmonics that should be concerned when identifying different instruments. The classification model based on attention network, which draws on the characteristics of human auditory attention, improves the recognition score of the main semiautomatic digitally played musical instruments and the overall recognition accuracy of all musical instruments. The two-level classification model is divided into a first-level classification model and a second-level classification model. The second-level classification model consists of three residual networks, which are separately semiautomatically trained to specifically identify strings, wind instruments, and percussion instruments. That is, the first-level classification model first performs the rough classification of the musical instrument family, and then the second-level classification model uses a special musical instrument family classification network to subdivide a certain musical instrument on the basis of the rough classification and finally summarizes the classification results. First, when extracting pitch features, this paper uses a filter bank with recursively set parameters to extract the primary features of audio, which reduces the number of parameters of the traditional end-to-end network and effectively reduces the risk of overfitting. Then, this paper introduces the constant Q transform in combination with the music theory knowledge of the twelve-average law. When extracting the constant Q transformation matrix of the audio, it is first transformed by each octave and then summarized to reduce the calculation time.

## 2. Related Work

In recent years, automatic classification of audio has also attracted increasing attention in related fields such as video retrieval and summarization, and content-based speech retrieval. Especially for solving general problems such as space-time information storage and parallel search, self-organized associative memory, self-organization of space-time data statistical description, and automatic knowledge acquisition from some interrelated activities, it shows unique capabilities. In video retrieval and summarization, it is found that simple visual features such as color, texture, motion vector, etc. do not reflect the content and structural semantics of videos well, while the extraction of more advanced visual semantic features is quite difficult [16].

Content-based speech retrieval mechanisms include keyword sporting, sub-word indexing, and continuous speech recognition in it [17], but they are all expensive, and the retrieval effect is relatively high and depends on the specific speech environment. If the audio is automatically classified to determine the sound environment, the recognition accuracy and efficiency can be improved. Pérez et al. [18] proposed a method to distinguish speech/music using energy, latent entropy, etc. as parameters and achieved a correct recognition rate of 90%. Xie et al. [19] proposed using Mel frequency scale cepstral coefficients, line spectrum pair parameters, and a classification modeling method to distinguish non-speech, music/non-music, and obtained 99.5% power u93% recognition, respectively. Deperlioglu et al. [20] adopted a multi-step unit sub-classification method for speech/music based on a simple decision tree; that is, each step determines the category of the audio according to one or more audio features and their values of 90%, 82% accuracy. Starting from the rhythm of the audio, Golub et al. [21] classified three kinds of audio: voice, music, and background, and obtained a 95% correct recognition rate. And the recognition accuracy rate was, respectively, 90.9% to 86.9%.

The article "Design of Semiautomatic Digital Creation System for Electronic Music Based on Recurrent Neural Network" was published in 2022. Journal: Comput Intell Neurosci.

However, the unit sub-classification model can only represent statistical characteristics such as mean and variance, while audio signal characteristics usually have temporal statistical characteristics [22]. For example, music generally has a rhythm or drum beat that reveals the theme, and in speech, voiced and unvoiced sounds often alternate. The unit-level model is less effective at identifying these features. Therefore, it is obvious that there are certain limitations to identify audio files only based on frequency domain characteristics. The neural network model is an ultra-large-scale nonlinear continuous-time adaptive information processing system. It is a method based on the discriminant model proposed on the basis of the results of modern neuroscience research. It reflects the basic characteristics of human brain function to a certain extent [23–26]. Through reasonable semiautomatic training of recurrent neural network, it can have strong discriminative ability.

## 3. Recurrent Neural Network Music Digital Creation

### 3.1. Eigenvalues of Recurrent Neural Networks

DenseBlock in recurrent neural network is a key component of DenseNet. DenseNet completes its network structure by stacking a large number of DenseBlocks. Dense connections add diversity to the input and improve efficiency. This is also a big difference between DenseNet and ResNet. This dense connection design makes DenseNet require fewer parameters than other ordinary recurrent neural networks, because there is no need to learn repeated features in DenseNet. At the same time, the connection between DenseBlocks adopts a simple connection, and a transition unit is added between the DenseBlocks. By controlling the compression parameter *θ* of the unit, the compactness of the model can be further improved and feature compression and dimension reduction can be provided, so that it can be easily semiautomated training and deep network structure.

(1) $$\begin{array}{c} u\left(x,y\right)=\left\{\begin{array}{c} \sum_{i=1}^{n}x\left(r,s\right)-\frac{\left|r_{i}-s_{i}\right|}{\left|t_{i}-s_{i}\right|},\\ \sum_{i=1}^{n}y\left(t,s\right)-\frac{\left|r_{i}+s_{i}\right|}{\left|t_{i}-s_{i}\right|}. \end{array}\right. \end{array}$$

In a feedforward network, neurons are arranged in layers, which can be a single layer or a multi-layer, but usually there are at most two layers; the transmission of data is passed from front to back. In the regression network, the neurons are arranged in layers, and the data is forwarded internally, but the results of the entire network can be fed back to the first layer, and through comparison, the connection weights between the layers can be corrected. In essence, it is to find an optimal normalization function to match the elements in two template sequences of different lengths one-to-one. Different application scenarios may have different mathematical expressions to characterize similarity or distortion. In this paper, the similarity of two element points on the template sequence is characterized by comparing the Euclidean distance of the two feature vectors in Figure 1.

The article "Design of Semiautomatic Digital Creation System for Electronic Music Based on Recurrent Neural Network" was published in 2022. Journal: Comput Intell Neurosci.

The twelve equal temperament shows that each octave is divided into twelve semitones, taking the sound name A as an example, and there will be a semitone named A in each octave, and their corresponding fundamental frequencies are different (later). One is twice the previous one, the set of all semitones with A as the sound name is called sound level A, and all its energy is accumulated to get the energy of sound level A.

(2) $$\begin{array}{c} v\left(t,s\right)=\sum_{t,s}x\left(t,s-1\right)-\sum \mathrm{hermiter}\left(t-s\right)x\left(t,s-t+1\right). \end{array}$$

The same is true for other semitones, so a feature vector representing the energy distribution of 12 pitch levels is obtained, which is called a chrominance (Chrome-Pitch) feature, or a map feature. Based on this idea, this paper adopts a method to extract the spectral features of audio.

### 3.2. Digital Audio Extraction

The characteristics of the digital audio filter bank are as follows: there are 13 triangular filters with a center frequency below 1000 Hz, and their center frequencies are linearly distributed, separated by 66.666667 Hz; there are 27 triangular filters with a center frequency above 1000 Hz, and their centers in the frequencies are distributed in a proportional series with a scale of 1.0711703. The low-frequency cutoff frequency of the lowest frequency filter is 133.33333 Hz. The low-frequency cutoff frequency of the last filter is equal to the center frequency of the previous filter. After the frequency domain signal passes through these 40 triangular filters, the linear frequency scale is converted into a Mel frequency scale.

(3) $$\begin{array}{c} \left\{\begin{array}{c} \exp\;x\left(m,s\right)w\left(m,t\right)=\frac{w\left(m,t\right)}{x\left(m,s\right)},\\ \exp\left(\text{iwm}-\text{jwm}\right)=\frac{\exp\left(\text{iwm}-\text{jwm}\right)}{\exp\left(\text{iwm}-\text{jwm}\right)}. \end{array}\right. \end{array}$$

After using the additional momentum method, if the semiautomatic training of the network reaches the local minimum value, due to the influence of the additional momentum, the network model will continue to search for the minimum value, which may jump out of the local minimum value until the global minimum value is found. However, during semiautomatic training, due to the difference of initialization parameters, the neural network model will stop semiautomatic training occasionally when the error reaches the local minimum value. The strength of music is the strength of the sound. In the score, the velocity is usually marked by the Italian musical term, P for weak, F for strong; from weakest to strongest can be divided into a dozen levels, marked above the notes. The changes in intensity are very detailed and complex. When playing, the performer will make specific and detailed changes according to their own understanding of the music under the guidance of the score.

The article "Design of Semiautomatic Digital Creation System for Electronic Music Based on Recurrent Neural Network" was published in 2022. Journal: Comput Intell Neurosci.

The key to the exponential smoothing method is the selection of the smoothing coefficient. The value of Figure 2 is easily affected by some subjective factors. Different values will lead to a large difference in the prediction error. Therefore, it is necessary to select an appropriate smoothing coefficient to minimize the prediction error of the prediction model. Generally, the heuristic method is used to determine the value of the smoothing coefficient when the quadratic exponential smoothing method is used for prediction. Assign different smoothing coefficients to experiment, and calculate the sum of squares of errors between the algorithm output and the actual output.

(4) $$\begin{array}{c} \left\{\begin{array}{c} \exp\left(\text{jwn}-\text{rwm}\right)=x\left(m,s\right),\\ \mathrm{derfert}\left(\text{shift}-\text{mwr}\left(x\right)-x\right)=\exp\left(\text{iwm}-\text{jwm}\right). \end{array}\right.. \end{array}$$

The smoothing coefficient with the smallest sum of squares is the best smoothing coefficient. When the smoothing coefficient is close to 1, the influence of observations farther away from the predicted value decreases more rapidly. When the smoothing coefficient is closer to 0, the influence of observations farther from the predicted value on the predicted value decreases more slowly. Therefore, when the data is relatively stable, the smoothing coefficient is relatively close to 0; when the time series fluctuates more severely, the smoothing coefficient is closer to 1.

The article "Design of Semiautomatic Digital Creation System for Electronic Music Based on Recurrent Neural Network" was published in 2022. Journal: Comput Intell Neurosci.

### 3.3. Numerical Analysis of Recurrent Networks

After applying the local connection of the recurrent network, the number of parameters is greatly reduced, but the number of parameters is still large. To solve this problem, the concept of weight sharing came into being. Weight sharing is based on the assumption that if a feature is valuable at (*x*1, *y*1), it should also be valuable at (*x*2, *y*2). Other parts are the same.

(5) $$\begin{array}{c} \left\{\begin{array}{cc} \frac{f^{-1}\left(x-y\right)}{\text{fertec}\left(x\right)-\text{fertec}\left(y\right)}, & x>y,\\ 1-\frac{1}{\text{fertec}\left(x\right)-\text{fertec}\left(y\right)}, & x<y. \end{array}\right. \end{array}$$

Therefore, for the aforementioned example, this paper can force the parameters contained in 10,000 music power units to be consistent; then under this premise, the number of parameters is reduced to 10 × 10 × 3 + 1 = 301. This paper uses the same parameters to slide the whole music from left to right and from top to bottom and calculate the summation of matrix products (recursive operation), so this part of the parameter matrix is called a recurrent neural network kernel in this paper. In order to extract different types of features, multiple recursive kernels are usually set in a recursive unit to ensure the diversity of features.

(6) $$\begin{array}{c} \text{feteact}\left(x,y\right)=\frac{f^{-1}\left(\text{fertec}\left(x\right)-\text{fertec}\left(y\right)\right)}{f^{-1}\left(\text{fertec}\left(x\right)+\text{fertec}\left(y\right)\right)}. \end{array}$$

From the perspective of MIDI format analysis, there are also velocity velocity, note number NoteNumber, and syllable number BarNumber in MIDI information that can be extracted. The speed refers to the speed of music, which is divided into slow, fast, medium, and gradual, gradually slowing down, etc.; the number of notes NoteNumber refers to the number of notes contained in the entire piece of music; the number of syllables BarNumber refers to the number of syllables contained in the entire piece of music. If the error function value is indeed reduced, then it means that the learning rate value selected by the algorithm. If it is too small, the learning rate can be appropriately increased on the basis of the original; on the contrary, if the error function does not decrease, it means that the learning rate is overregulated. At this time, the value of the learning rate should be reduced until the system reaches convergence.

The article "Design of Semiautomatic Digital Creation System for Electronic Music Based on Recurrent Neural Network" was published in 2022. Journal: Comput Intell Neurosci.

The electrical impulse signal as shown in Figure 3 is transmitted from the music power unit through the axon, first reaching the axon terminal; at this time, the vesicles in it are changed to release neurotransmitters, which enter through the synaptic gap into the branches of another musical power unit. It can accept a set of input signals from other music power units in the system, each input corresponds to a weight, and the weighted sum of all inputs determines the activation state of the music power unit. Suppose *n* input signals are represented by *x*, respectively, their corresponding connection weights are in turn *y*, and the expected output signal is *y*(*f*). All inputs and corresponding connection weights constitute input vector *x* and connection weight vector *W*, respectively.

### 3.4. Analysis of Internet Music Power Spectrum

The idea that recurrent neural networks obtain local correlations in space by applying local connections is intuitively consistent. When people have cognition to the outside world, they also go from part to whole, and for information such as music, the local correlation is more obvious. Therefore, in the recurrent neural network, each music power unit only needs to be connected to a small part of the music power unit of the previous unit after applying local connection. This semiautomatic digital operation greatly reduces the number of model parameters.

The ability of a single-stage network is very limited. Properly increasing the number of network units (the number of hidden units) is a way to improve the neural network's cognitive ability, which also simulates some parts of Figure 4 to a certain extent hierarchical features.

(7) $$\begin{array}{c} \text{fert}\left(e\left(x\right),t\right)=\int \text{fer}\left(\exp\left(t\right),x\right)*\;\exp\left(2\text{pix}\left(x\right)\right)\text{d}x\text{d}t-1. \end{array}$$

The number of hidden units in the network and the number of music power units in each hidden unit are problem-related. The current research results are also difficult to give a functional relationship between them and the type of problem and its size. The number of music power units of the output unit is determined as follows: the objects to be distinguished are divided into three categories: speech, music, and mixed sounds, so the number of music power units of the output unit is determined as 3. The number of hidden unit music power units takes half of the sum of the number of input and output unit music power units, namely, (13 + 3)/2 = 8.

The article "Design of Semiautomatic Digital Creation System for Electronic Music Based on Recurrent Neural Network" was published in 2022. Journal: Comput Intell Neurosci.

## 4. Design of the Semiautomatic Digital Creation System for Electronic Music Based on Recurrent Neural Network

### 4.1. Recurrent Neural Network Coding

The paper uses Vc++ to implement the algorithm and selects 200 MIDI songs to test the positioning of the main track, of which 194 have found the main track correctly, 6 have not been found, and the accuracy rate is 97%, basically reaching system requirements. Looking at these 6 songs, we found that they all have the characteristics of the main melody beating violently, making the pitch stability not as good as some accompaniment tracks. There is a dual relationship between the time domain signal and the frequency domain signal, which can be converted to each other. Fourier transform can transform complex time-space signals into frequency signals and then use simple spectrum analysis to complete the complex analysis of the original signal, and the transformation process uses the information of the entire time domain of the signal to calculate the spectrum value of each frequency component. In fact, the signal is complex and changeable, and the existence time of each frequency component is not necessarily as long as the entire signal, but the global transformation method of the Fourier transform will solve the problem

(8) $$\begin{array}{c} \frac{1-\int \text{fer}\left(\exp\left(t\right),x\right)\text{d}x\text{d}t}{\int \exp\left(2\text{pix}\left(x\right)\right)\text{d}x\text{d}t}*\frac{1}{\exp\left(2\text{pix}\left(x\right)\right)}=\emptyset . \end{array}$$

After analysis, it can be seen that when building a neural network model for the artist's song audition, the number of input music power units is 34, the number of output music power units is 1, and the number of hidden unit music power units is 8 and only one music power unit. Build this algorithmic model and predict the artist's daily song audition volume from August 1, 2019, to August 30, 2019. When using the neural network algorithm for prediction, the neural network can simulate the development trend of things to a certain extent, and even some small data fluctuations can be predicted by the algorithm. The prediction error mainly depends on the semiautomatic training effect of the semiautomatic training data of the neural network model, the selection of Table 1, the number of hidden unit neurons, etc.

The experimental results are taken from the average of the 10-fold cross-validation results. Considering that the length of the audio sample is different, the extracted audio feature size is also inconsistent. In addition, its size is also very large. Taking the setting of this paper as an example, the Mel power spectrum feature size of a single sample reaches 128 × 644; if all samples are considered, the size of all samples is 900 × 82432 when they are combined into a matrix for semiautomatic training, so it is difficult to directly use these features as the input of the classification model. Before the semiautomatic training, this paper normalizes the semiautomatic training data, so that the semiautomatic training data has a mean of 0 and a variance of 1 in each feature dimension.

(9) $$\begin{array}{c} \text{for}\left\{m>n>f\left(m,n\right)-1\right\}⟶\left\{\begin{array}{c} \text{fertc}\left(m,n\right)<f\left(m\right)-f\left(n\right),\\ f\left(m\right)+f\left(n\right)<\frac{1}{\text{fertc}\left(m,n\right)}. \end{array}\right. \end{array}$$

After the standard normalization, this paper also uses principal component analysis which is used to reduce the dimensionality of the features and retain 99% of the variance on the original dataset. The semiautomated numerical operation of principal component analysis is only used for classifiers other than XGBoost.

The article "Design of Semiautomatic Digital Creation System for Electronic Music Based on Recurrent Neural Network" was published in 2022. Journal: Comput Intell Neurosci.

### 4.2. Reconstruction of Online Music Classification

In this paper, we write some related functions for semiautomatic training of classification reconstruction. For example, in order to classify audio, it is necessary to apply the sample input vector and ideal output vector to the semiautomatic training. In this paper, a TotalFeature (NUM) function is written to obtain the feature vector and form the matrix input as the input vector of the sample and at the same time generate a matrix target as the ideal output vector of samples. Then design a function CreateAndFrain-NN, according to the previously obtained and preprocessed sample input vector and ideal output vector, call newff to establish a feedforward BP network, and set up the activation function and training method, then initialize the network, and call the frin function to semiprocess the network.

(10) $$\begin{array}{c} \log\left(\text{imagert}\left(x,t\right)-\frac{1-x}{300}\right)-1200\;\log\left(e\left(x\right)-x\right)\left(1-\frac{1-x}{300}\right)=0. \end{array}$$

The function contains pitch information. The found pitch information is stored in the corresponding array according to the track. If the newly found pitch does not have a corresponding array, a new array is created. A formula for defining the equal-height Mel filter is shown in it. The Mel power spectrum can be obtained by passing the Hertz power spectrum through a set of Mel filters.

(11) $$\begin{array}{c} \frac{\text{fermertc}\left(n-1/f\left(\text{signal}\left(t\right)-t\right)\right)}{\text{signal}\left(t\right)}-{\text{siganle}}^{-1}\left({\text{mel}}^{-1}\left(t\right)-1\right)=\frac{1}{1+\text{signal}\left(t\right)}. \end{array}$$

The Bach10 dataset is a polyphonic (multi-voice) music dataset that serves as a standard dataset for a variety of music research problems, such as multi-tone estimation and tracking, audio score calibration, source separation, etc. The dataset includes ten large-scale choral works by J.S. Bach, each of which contains four monophonic parts, soprano, alto, tenor, and bass. The semiautomated digital performance instruments used for the audio recordings of each single part were violin, clarinet, saxophone, and bassoon.

The article "Design of Semiautomatic Digital Creation System for Electronic Music Based on Recurrent Neural Network" was published in 2022. Journal: Comput Intell Neurosci.

The dataset provides the quartet chorus works of Figure 5, and this paper can generate more recordings with different polyphony by exploring the combination of different voices in each work. For each choral piece, the maximum number of audio records that can be produced is 15, containing four monophonic parts, six duets, four trios, and one quartet. These new recordings have the same semiautomated digital performance dynamics as the original recordings, providing instrument recognition algorithms with samples of multi-instrument semiautomated digital performance test data at different polyphony.

### 4.3. Semiautomated Numeric Symbol Mapping

IDI music has 3 modes: single-track mode, multi-track sync mode, and multi-track asynchronous mode. In the single-track mode, the characteristics of the music are all included in this track, and the results of analyzing this track are accurate for sentiment classification. Through the local connection and weight sharing of recursive units and the downsampling process of pooling units, the recurrent neural network greatly reduces the number of parameters and increases the translation invariance to a certain extent. High-dimensional matrix input, such as music data, is input as 100 × 100 × 3 (width × height × channels). When using the Mel power spectrum as input features, logistic regression and random forest models using L2 regularizers showed better classification results. Considering the data scale of the GTZAN dataset itself and the maximum difference of about 2% in the classification accuracy of the two audio features in Figure 6 on all classification models, we believe that these two features have similar effects on the classification effect.

The dataset consists of 122 songs, 108 of which include melody annotations. The remaining 14 songs have no discernible melody and are therefore not suitable for melody extraction, but are included in the dataset because they can be used for other applications including instrument identification, source separation, and automatic mixing. Most songs were recorded in professional studios and mixed by experienced engineers (30 songs from various independent artists, 32 songs at Dolan Studios, 25 songs at Weathervane Music Studios, and Music Delta Studio recorded 35 songs).

(12) $$\begin{array}{c} y\left(f\left(t\right),t\right)=\langle \begin{array}{c} \int_{-1}^{1}\text{wermet}\left(t-x\right)x\left(t\right)\text{d}x\text{d}t-1,\\ \frac{\int 1-x\left(t\right)\text{d}x\text{d}t}{\int x\left(t-1\right)\text{d}x\text{d}t}. \end{array} \end{array}$$

Detuned-mode oscillators outperform critical-mode oscillators in a variety of networks. This can be attributed to the hijacking phenomenon mentioned above. The change of the tempo of the music piece can be regarded as the hijacking process among the local oscillator groups in the network, in order to better realize the beat tracking. In local areas where strong resonance occurs, the oscillators will exhibit similar frequencies. As the stimulation frequency changes, this local region can follow its changes, moving the resonance region along the frequency gradient. On this basis, in the semiautomatic training process, this paper randomly selects the starting point for each sample and sequentially intercepts multiple samples of the same length. This makes the model in this paper actually observe only about 7.5 seconds of audio information for each semiautomatic training sample during semiautomatic training, instead of the full-length 30-second sample, so that the model has more data for semiautomatic training.

The article "Design of Semiautomatic Digital Creation System for Electronic Music Based on Recurrent Neural Network" was published in 2022. Journal: Comput Intell Neurosci.

## 5. Application and Analysis of the Electronic Music Semiautomatic Digital Creation System Based on Recurrent Neural Network

### 5.1. Recurrent Neural Network Data Decoding

The music power unit contained in the recurrent neural network data constitutes the input unit of the entire neural network, which is usually used to receive input signals from the outside world. The music power unit contained in the red box constitutes the output unit of the neural network, which is used to provide the neural network's perception and processing results of the input signal, and the result is usually in the form of a number (regression model) or a vector (classification). All units except input and output units are called hidden units.

(13) $$\begin{array}{c} \mathrm{dertal}\left(i,j\right)=\left\{\begin{array}{cc} 0, & i>j,\\ 1-\frac{i}{j}-1-\frac{j}{i}-1, & i<j. \end{array}\right. \end{array}$$

The type part of the data block is the 4-byte ASCII code MTrk, which indicates that the block is the data block of the MIDI file; the second part of the length indicates the length of the block; the third part is the main content of the MIDI file, which contains many <delta-time>. The sequence of <time><event>, the pitch, length, dynamics, etc. of the music are hidden in it. Note that rap music and most synthesized songs do not have melody annotations. A total of 105 of the 122 songs in the dataset are full-length songs, most of which are 3 to 5 minutes in length. Most of the sub-1 minute recordings were created by Music Delta Studios.

The article "Design of Semiautomatic Digital Creation System for Electronic Music Based on Recurrent Neural Network" was published in 2022. Journal: Comput Intell Neurosci.

If the ensemble is highly biased, that is, for the same input in Figure 7, all the networks in the ensemble give the same or similar outputs, at this time the degree of difference of the ensemble is close to 0, and its generalization error is close to the generalization error of each network of weighted average of the errors. Conversely, if each network in the ensemble is independent of each other, the degree of difference in the ensemble will be large, and the generalization error will be much smaller than the weighted average of the generalization errors of each network. Therefore, in order to enhance the generalization ability of neural network ensemble, it is necessary to make the errors of each network in the ensemble as uncorrelated as possible.

### 5.2. Electronic Music Semiautomatic Digital Creation Simulation

The simulation implementation is based on the following reasons: (1) different musical instruments can semiautomatically play different numbers of notes, and each note corresponds to a pitch frequency, also called the fundamental frequency (note that the fundamental frequency is a physical quantity, and the pitch is a musical perception concept, often used equivalently in music computing literature), such as a piano that can emit 88 notes of different fundamental frequencies; (2) different musical instruments have different pitch ranges pitch range is from 27 Hz to 4.1 kHz; (3) it helps to capture the harmonic structure. The harmonic is the integer multiple frequency corresponding to the fundamental frequency. If the fundamental frequency is found, the position of the harmonic can be quickly captured and the structure of the harmonic can be obtained; (4) it is beneficial to locate the start and end frames and the end frame, and the fundamental frequency can be captured, indicating that it is a non-stationary sound, and it is easy to judge the start and end of the audio signal. The stability of the pitch can reflect the intensity of mood swings. We can find the average pitch of the music, which is represented as a horizontal line on the score, and all the notes float up and down on this horizontal line. The fluctuation is small; that is, the pitch is relatively stable, and the emotional fluctuation of the music is small. The lyrical narrative music often has this feature.

The article "Design of Semiautomatic Digital Creation System for Electronic Music Based on Recurrent Neural Network" was published in 2022. Journal: Comput Intell Neurosci.

Since different instruments can semiautomatically play the notes digitally, the specific fundamental frequencies and numbers in Figure 8 are not exactly the same (88 for piano, 41 for cello, 35 for trombone, 34 for trumpet, etc.), and a certain time frame is determined.

(14) $$\begin{array}{c} y\left(t,t-1\right)=\sqrt{\frac{2-t}{1-t}}\sum \frac{t\left(n\right)-T\left(n\right)}{t\left(n\right)-T\left(n\right)-1}-1. \end{array}$$

The notes played by the upper semiautomated numbers and their pitch frequencies can differentiate some instruments to a certain extent. It shows the corresponding pitch frequencies (unit: Hz) of the 88 notes that the piano can play digitally in a semiautomatic manner. The gray background represents the lowest and highest notes.

If the neural network model has been semiautomated training and is in a stable state, but a new set of semiautomatic training data needs to be learned, then the weights and thresholds in Table 2 are not suitable for the original semiautomatic training. The neural network model is not suitable for the current situation, and the original semiautomatic training data can only be combined with the new semiautomatic training data for semiautomatic training. After preprocessing semiautomatic digital operations such as framing the synthesized audio and the original audio, combined with the note endpoint detection algorithm, perform the above three steps to obtain the map features of the note fragment, add the values in each semitone of the same name, and finally get one for each frame.

### 5.3. Example Application and Analysis

The competition data in the Ali Music Trend Prediction Contest used in the experiment in this paper is derived from the semiautomatic digital music operation record data of real users in the Ali music platform application. This data records a large number of semiautomated digital manipulation (audio, download, and favorite) recordings of all songs of a hundred artists from March 1, 2019, to August 30, 2019. The data consists of two parts: the data that records the song, and the record of the semiautomated digital manipulation of the song by the user. During the period, the semiautomatic digital operation (audio listening, downloading, and collecting) records of 26,958 songs of the 100 artists included a total of 15,884,087 user semiautomatic digital operation records.

Therefore, before conducting the experiment, it is necessary to screen out some artists who need algorithm prediction from many artists. The factors affecting the audition volume of an artist's songs are mainly related to the total number of the artist's recent song audition and the recent audition volume of some of the artist's songs. The establishment of samples is divided into two steps. This article first selects 150 works that are enough to cover all emotions from a large number of MIDI music libraries and then spends 3 months to invite 20 people including classmates, family members, and friends to listen to each song and listen to it, the results are recorded in the form of questionnaires, and the emotions of each work in the minds of most people are determined.

The article "Design of Semiautomatic Digital Creation System for Electronic Music Based on Recurrent Neural Network" was published in 2022. Journal: Comput Intell Neurosci.

This paper uses a recurrent neural network to perform the 5 × 10-fold cross-validation in Figure 9 on the ISMIR2004 dataset. Compared with the GTZAN dataset, the ISMIR2004 dataset is more irregular. The number is unevenly distributed and it is a very unbalanced dataset. In the semiautomatic training process and verification process, in order to ensure the consistency with the semiautomatic training parameters of the GTZAN dataset, all samples whose duration is less than 30 seconds at the sampling frequency of 22050 Hz are excluded in this paper. According to statistics, after the semiautomatic digital operation is eliminated according to the aforementioned rules, the original training set, development set, and evaluation set are, respectively, eliminated 5, 5, and 3 samples. In the following design, six emotion feature vectors are the input of the neural network, and one type is the output of the neural network. Among the 150 pieces of music, 50 pieces of music that can cover the emotional space of music are selected as the training samples of the neural network, and the remaining 100 pieces of music are left as the test of the system. The highest classification accuracy rate in 5 × 10-fold cross-validation is 87.68%, and the average accuracy of 5 × 10-fold cross-validation is 87.11%. The number of music genre categories in the ISMIR2004 dataset is 6, which is 4 fewer than the GTZAN dataset. As can be seen, the RNN is lacking in classification on the Rock/Pop category, an observation that is similar to the results on the GTZAN dataset.

## 6. Conclusion

This paper implements a semiautomatic digital classification system for music genres based on recurrent neural networks and verifies the effectiveness and advancement of recurrent neural networks through this system. This paper designs new model architecture for music genre classification. It introduced and used DenseNet proposed in the frontier research in the field of computer vision as the basic model structure, combined with the idea of the proposed inception structure and designed and implemented a new recurrent neural network architecture and recurrent neural network; the model uses audio clip-based prediction method greatly. Experiments show that the model outperforms multiple classification models using recursive features designed by domain experts combined with classical machine learning models and compares the advantages of recurrent neural networks compared to multiple variant models. According to the different values of these two dimensions, the emotional space is divided into 9 regions, and the 9 regions are described with reference to the adjectives of Hevner's emotional circle. After the model is semiautomatically trained on a large dataset containing hundreds of thousands of audio samples, its classification effect on other standard data sets has been greatly improved, and the extracted features have good generalization ability to improve classification performance in other tasks.

The article "Design of Semiautomatic Digital Creation System for Electronic Music Based on Recurrent Neural Network" was published in 2022. Journal: Comput Intell Neurosci.

## Figures and Tables

**Figure 1:** Similarity distribution of eigenvalues of recurrent neural network.

**Figure 2:** Recursive network digital audio extraction distribution.

**Figure 3:** Recursive network digital topology.

**Figure 4:** Distribution of network elements in the network music power spectrum.

**Figure 5:** Online music classification and reconstruction test data.

**Figure 6:** Polar distribution of semiautomatic digital symbol mapping.

**Figure 7:** Electronic music semiautomated digital dependencies.

**Figure 8:** Electronic music semiautomation fundamental frequency distribution.

**Figure 9:** Distribution of semiautomated digital operations in online music.

**Table 1:** Recurrent neural network coding.

Recurrent unit	Development parameter	Network coding	Network weight
10	V-net	Code data	0.87
20	Cnn-test	The semiautomatic training	0.40
30	*F*(*x*)-text	Test data	0.45
40	Algorithm-t	The neural network	0.77
50	Cet-tain	All samples are considered	0.43
60	Case-line-t	Training data	0.11

**Table 2:** Recurrent neural network pitch frequency analysis algorithm.

Recurrent neural network content	Pitch frequency analysis algorithm
Input pitch frequency network: *fertc*(*m*, *n*)	After preprocessing semiautomatic
Input frequency network: *f*(*m*) − *f*(*n*)	Steps to obtain the map *x*(*t*)*dx* *dt*
Input pitch network: *f*(*m*)+*f*(*n*)	Digital operations such as *f*(*m*)
Input case pitch frequency network: exp(2*pix*(*x*))	Combined with the note
Plt.figure (figsize = (8, 4))	Framing the synthesized audio
Ax1 = plt.subplot (111, projection = 'polar')	Features of the note fragment
Ax1.set_title (“spot fish”)	log(*e*(*x*) − *x*)
Ax1.set_rlim (0, 12)	Perform the above three
Bar = ax1.bar (theta)	Data, alpha = 0.5
Data = np.random.randint (1, 10, 10)	Endpoint detection algorithm
Theta = np.arange (0, 2 ∗ np.pi, 2 ∗ np.pi/10)	*wermet*(*t* − *x*)

The article "Design of Semiautomatic Digital Creation System for Electronic Music Based on Recurrent Neural Network" was published in 2022. Journal: Comput Intell Neurosci.

## Data Availability

The data used to support the findings of this study are available from the corresponding author upon request.
